RETRACTED

# Influence of Adenoid Hypertrophy on Malocclusion and Maxillofacial Development in Children

**DOI:** 10.1155/2022/2052359

**Published:** 2022-07-07

**Authors:** Liping Zhang, Hui Liu

**Affiliations:** ^1^Department of Stomatology, Zhuji People's Hospital, Zhuji 311800, Zhejiang Province, China; ^2^Operating Room, The First Affiliated Hospital of Hunan Traditional Chinese Medical College, Zhuzhou 412000, Hunan Province, China

## Abstract

**Objective:**

To investigate the effect of adenoid hypertrophy on malocclusion and maxillofacial development in children.

**Methods:**

Total of 102 children with malocclusion or maxillofacial dysplasia admitted to our hospital from March 2017 to June 2020 were selected as the research subjects. All children were divided into a control group (50 cases with adenoid hypertrophy) and an observation group (52 cases without adenoid hypertrophy) according to the presence or absence of adenoid hypertrophy. The incidence of malocclusion was compared between the two groups, and lateral cranial radiographs were taken in both groups to measure and compare the malocclusion angle, jaw angle, and jaw length indexes between the two groups.

**Results:**

The incidence of malocclusion in the observation group (71.15%) was higher than that in the control group (42.00%), and the difference was statistically significant (*P* < 0.05). The angle between the long axis of the upper central incisor and the nasal root point and the upper alveolar base point (U1-NA), the angle between the long axis of the lower central incisor and the nasal root point and the lower alveolar base point (L1-NB), the angle between mandibular plane and anterior cranial base plane (MP-SN), the angle between the long axis of upper central incisor and anterior cranial base plane (U1-SN), the angle between the long axis of lower central incisor and mandibular plane (L1-MP), the angle of *Y* axis, the overall height (N-Me), lower height (ANS-Me), overall height/back height (N-Me/S-Go), and lower height/overall height (ANS-Me/N-Me) values in the observation group were higher than those in the control group, while the mandibular length (Go-Gn) values in the observation group were lower than those in the control group (*P* < 0.05).

**Conclusion:**

Adenoid hypertrophy can increase the incidence of malocclusion in children and can also increase the steepness and overall height and lower height of the mandible, resulting in the lengthening of the facial shape and the development of the maxillofacial deformity.

## 1. Introduction

The dental and maxillofacial growth and development of children is a complex but coordinated and continuous process with great growth potential in the upper and lower jaws, which is influenced by a combination of genetic factors, behavioral patterns, and environmental factors [1, 2]. The adenoids, also known as pharyngeal tonsils, are also an important part of the pharyngeal lymphatic ring (Waldeyer's ring) and play an important immune-inducing role as a physiological defense mechanism of the body, against inhaled allergens and microorganisms [3, 4]. The adenoids are located at the top of the nasopharynx and the posterior pharyngeal wall, and when the adenoids or their surrounding lymphatic tissues are repeatedly stimulated by inflammation, this can lead to pathological hyperplasia of the adenoids, resulting in adenoid hypertrophy [5, 6]. When pathological hyperplasia of adenoids occurs, it is highly likely to cause a variety of diseases such as otitis media, inflammation of the lower respiratory tract, and even sleep apnea [7, 8].

RETRACTED

Adenoid hypertrophy can lead to blockage of the already narrow nasopharynx in children affecting breathing, when the child's nasal airway is blocked and ventilation is reduced, causing a physiological neuromuscular feedback effect and passive stretching of the head and neck muscles, and then, open-mouth breathing occurs [9, 10]. Long-term open-mouth breathing often tends to trigger abnormal neuromuscular activity, causing relative body position changes in the maxillofacial muscles, resulting in abnormal development of the upper and lower jaws, which affects the normal development of the child's maxillofacial structures and eventually leads to imbalance or even deformed development of the maxillofacial morphology [11, 12]. Bandyopadhyay and Slaven [13] found that abnormalities in the anatomical structures adjacent to the upper airway or multiple lesions can cause open-mouth breathing, such as tonsillar hypertrophy, adenoid hypertrophy, allergic rhinitis, nasal septal deviation, and turbinate hypertrophy nasal stenosis, but it is now generally accepted that adenoid and tonsillar hypertrophy are the most important causes of open-mouth breathing in childhood. The aim of this study was to investigate the effects of adenoid hypertrophy on malformation and maxillofacial development in children. The details are reported in this study.

## 2. Information and Methods

### 2.1. General Information

One hundred and two children with malocclusion or maxillofacial developmental abnormalities admitted to our hospital from March 2017 to June 2020 were selected for the study, including 55 males and 47 females, aged 3–12 years, with an average age of (8.01 ± 2.09) years. Inclusion criteria were as follows: all lateral cephalometric films were performed, no history of orthodontic treatment, and no other congenital diseases. Exclusion criteria were as follows: history of adenoidectomy; history of ear, nose, and throat related diseases; and those with upper respiratory tract infections.

RETRACTED

All children were grouped according to the presence or absence of adenoid hypertrophy: control group (50 cases): no adenoid hypertrophy, maximum adenoid thickness (A)/nasopharyngeal cavity width (N) value <0.71; observation group (52 cases): with adenoid hypertrophy, A/N value ≥0.71. There were 26 boys and 24 girls in the control group, aged 3–12 (7.86 ± 2.04) years. In the observation group, there were 29 boys and 23 girls, aged 5–12 (8.15 ± 1.96) years. The general data of the children in the two groups were compared, and the differences were not statistically significant (*P* > 0.05). The study was approved by the ethics committee of our hospital, and the families of the children gave their informed consent and signed the informed consent form.

## 3. Research Methodology

Referring to the literature [9], all children were classified into normal, An I, II, and III malocclusions, and the incidence of jaw deformity was counted. All children had lateral cephalometric films taken by the same physician using the Planmeca Proline XC system (Planmeca, Finland), with the child in a natural head position, no deflection, upper and lower lips closed naturally, no swallowing, and relaxed facial muscles. The measured images were transferred to the WinCeph 8.0 software, and all indicators were measured by the same physician, and each indicator was measured three times, and the final average was taken as the study data. Measurements include the angle between the NPo of the face plane and the SN of the anterior cranial base plane (NPo-SN), angle (U1-NA) between the long axis U1 of the upper central incisor and the line connecting the nasal root point and the seat point of the upper tooth groove, angle between the long axis of the lower central incisor L1 and the line connecting the nasal root point and the seat point of the lower tooth groove (L1-NB), angle between the long axis L1 of the lower central incisor and the Gn-Me angle in the mandibular plane (IMPA), subspinale plane angle (SNA), supramental plane angle (SNB), AB plane angle (ANB), angle between the mandibular plane MP and the anterior skull base plane SN (MP-SN), angle between the long axis of the upper central incisor U1 and the anterior cranial base plane SN (U1-SN), angle between the long axis of the lower central incisor L1 and the mandibular plane MP (L1-MP), angle between the line connecting the butterfly saddle point and the chin vertex and the orbital ear plane (*Y*-axis angle, SGn-FH), vertical distance between nasal root point and subchin point (N-Me), distance from the anterior nasal spine to the point under the chin (ANS-Me), vertical distance between the point of the butterfly saddle and the point of the mandibular angle (S-Go), N-Me/S-Go, ANS-Me/N-Me, and length of the corpora mandibulae (Go-Gn).  Figure 1 shows the details.

RETRACTED

### 3.1. Statistical Methods

SPSS 22.0 software was applied for processing, and the experimental data measurement data were expressed as mean ± standard deviation ($\bar{x}$ ± *s*), and the *t*-test was used for two-comparison analysis. Count data were expressed as (%), and the *χ*^2^ test was used. The test level was *α* = 0.05, and *P* < 0.05 was considered a statistically significant difference.

## 4. Results

### 4.1. Comparison of the Prevalence of Malocclusion between the Two Groups

In the control group, there were 10 cases of angle class I, 7 cases of angle class II, and 4 cases of angle class III, with a total of 21 cases of malformation, and the total incidence was 42.00% (21/50). In the observation group, there were 18 cases of angle class I, 11 cases of angle class II, and 8 cases of angle class III, totaling 37 cases of malformation, with a total incidence of 71.15% (37/52). The incidence of malformation in the observation group was higher than that in the control group (*P* < 0.05), as given in Table 1.

### 4.2. Comparison of Misshapen Angle Indexes between the Two Groups

He U1-NA and L1-NB values in the observation group were significantly higher than those in the control group (all *P* < 0.05); the differences in NPo-SN and IMPA between the two groups were not statistically significant (all *P* > 0.05), as shown in Figure 2.

### 4.3. Comparison of Jaw Angle Indexes between the Two Groups

The MP-SN, U1-SN, L1-MP, and *Y*-axis angle values were higher in the observation group than in the control group (all *P* < 0.05). There was no statistically significant difference in the comparison of SNA, SNB, and ANB between the two groups (all *P* > 0.05), as shown in Figure 3.

### 4.4. Comparison of Jaw Bone Length Indexes between the Two Groups

The N-Me, ANS-Me, N-Me/S-Go, and ANS-Me/N-Me values in the observation group were higher than those in the control group, and the Go-Gn values were lower than those in the control group (all *P* < 0.05); the difference between the S-Go values of the two groups was not statistically significant (*P* > 0.05), as shown in Figure 4.

## 5. Discussion

Maxillofacial growth and development in children are determined by a combination of genetic and environmental factors, with genetic factors playing an important role and environmental factors not being neglected. Maxillofacial growth occurs mainly during childhood and shows two growth spurts, the first between 5 and 10 years of age (the period of change from milk teeth to permanent teeth) and the second between 10 and 15 years of age [14], the first peak being also the age of high prevalence of physiological and pathological hypertrophy of the adenoids and/or tonsils. The adenoids are important immune organs in the nasopharynx, and inflammatory stimulation can lead to pathological hypertrophy and subsequent nasal congestion and nasosinusitis [15–17]. Adenoid hypertrophy occurs mostly in children and is the main cause of open-mouth breathing; adenoid hypertrophy can obstruct the upper airway in children, causing narrowing of the airway and respiratory distress; in order to better ventilate and enhance the respiratory effect, the body position of the bones and soft tissues of the maxillofacial region undergoes adaptive changes; this continuous change in body position can lead to an imbalance in the forces on the teeth and bones, resulting in abnormal development of the maxillofacial region [18]. As children are in the growth and development stage, their maxillofacial skeleton is not yet fully developed and is highly susceptible to breathing habits. Long-term open-mouth breathing can cause malfunction of the perioral muscles and soft tissues in children, which in turn affects the normal development of the child's maxillofacial skeleton and is more likely to form malformations [19, 20].

RETRACTED

The results of this study showed that the incidence of malocclusion was higher in the observation group than in the control group, indicating that adenoid hypertrophy can significantly increase the incidence of malocclusion in children. Analysis of the reasons for this is that the airway of children with adenoid hypertrophy is blocked, the breathing pattern changes, long-term open-mouth breathing will cause the palate to lift up, and the palate high arch phenomenon occurs after the impact of airflow; it will also cause changes in oral muscle activity; the function of the closed-lip muscle decreases, causing children to open their lips and expose their teeth, which breaks the balance between oral muscles and jawbone, leading to passive movement of teeth and protrusion of upper incisors, affecting the normal development of the jawbone, thus causing malocclusion [21]. Moreover, the results of this study showed that the U1-NA and L1-NB values in the observation group were higher than those in the control group, further indicating that adenoid hypertrophy promotes the occurrence of malocclusion in children.

The results of this study showed that the MP-SN, U1-SN, L1-MP, and *Y*-axis angle values were higher in the observation group than in the control group, indicating that the mandibles of children with adenoid hypertrophy underwent posterior rotation and the mandibles grew posteriorly, which is partially consistent with the results of previous studies [22, 23]. The results of this study showed that the N-Me, ANS-Me, N-Me/S-Go, and ANS-Me/N-Me values were higher in the observation group than in the control group, and the Go-Gn values were lower than in the control group, indicating increased mandibular steepness in children with adenoid hypertrophy. The reasons for this are that adenoid hypertrophy causes airway obstruction and narrowing of the upper airway in children, and at this time, the lower jaw needs to be extended forward to keep the airway open, plus open-mouth breathing causes the child's lower jaw to rotate back clockwise, increasing the steepness of the lower jaw and contributing to excessive vertical growth and development of the lower jaw, resulting in an elongated face and increased N-Me and ANS-Me [24, 25].

RETRACTED

In conclusion, adenoid hypertrophy can increase the incidence of malocclusion in children and also increase jaw steepness, N-Me and ANS-Me, leading to an elongated facial shape and causing malformations in jaw and facial development. Therefore, we should pay more attention to adenoid hypertrophy in children and actively prevent adenoid hypertrophy from causing poor jaw and facial development. In this experiment, it was difficult to collect children without malocclusion or abnormal maxillofacial development and their guardians who were unwilling to receive X-ray radiation, so normal children were not selected as a control group in this study, and the number of study subjects in this experiment was small and the conclusions were less convincing. In the long term, when the number of cases is sufficient, the results of this experiment will be demonstrated and the effects of different degrees of hypertrophy, duration, and age on maxillofacial growth and malocclusion in normal children and children with adenoidal hypertrophy will be further studied.

## Figures and Tables

**Figure 1:** Schematic diagram of imaging marker point measurement.

**Figure 2:** Comparison of misshapen angle indexes between the two groups. (a) NPo-SN. (b) UI-NA. (c) LI-NB. (d) IMPA. Compared with the control group, ^*∗*^*P* < 0.05.

**Figure 3:** Comparison of jaw angle indexes between the two groups. (a) SNA. (b) SNB. (c) ANB. (d) MO-NS. (e) UI-SN. (f) LI-MP. (g) S-Go-FH. Compared with the control group, ^*∗*^*P* < 0.05.

**Figure 4:** Comparison of jaw angle indexes between the two groups. (a) N-Me. (b) ANS-Me. (c) S-Go. (d) N-Me/S-Go. (e) ANS-Me/N-Me. (f) Go-Gn. Compared with the control group, ^*∗*^*P* < 0.05.

RETRACTED

**Table 1:** Comparison of prevalence of malocclusion between two groups (*n*, %).

Group	Class I	Class II	Class III	Total
Control group (*n* = 50)	10 (20.00%)	7 (14.00%)	4 (8.00%)	21 (42.00%)
Observation group (*n* = 52)	18 (34.62%)	11 (21.15%)	8 (15.38%)	37 (71.15%)
*χ* ^2^ value				8.833
*P* value				0.003

## Data Availability

The data used to support the findings of this study are available from the corresponding author upon request.

## References

[1] Oka S., Kawanabe H., Yamanobe S., Fukui K., Baba Y., Deguchi T. (2021). Relationship between olfaction and maxillofacial morphology in children with malocclusion. *Clinical and Experimental Dental Research*.

[2] Ribeiro R. A., Mattos A., Meneghim M. C., Vedovello S. A. S., Borges T. M. D., Santamaria M. (2021). Oral and maxillofacial outcomes in children with microcephaly associated with the congenital Zika syndrome. *European Journal of Orthodontics*.

[3] Calvo-Henriquez C., Branco A. M., Lechien J. R. (2021). What is the relationship between the size of the adenoids and nasal obstruction? A systematic review. *International Journal of Pediatric Otorhinolaryngology*.

[4] Yi X.-L., Yao L.-Y., Zhao P.-F., Yuan X.-Y., Wang Z.-C. (2021). Development patterns of adenoids in Chinese children without sleep-disordered breathing: a retrospective magnetic resonance imaging study with consecutive age groups. *Chinese Medical Journal*.

[5] Liu J. L., Li S. H., Cai Y. M. (2021). Automated radiographic evaluation of adenoid hypertrophy based on VGG-lite. *Journal of Dental Research*.

[6] Machado A. S., Silva A., Coutinho M., Sousa C. A. (2021). Platelet counts and adenoid hypertrophy: a neglected relationship. *Minerva Pediatrica*.

[7] Pachêco-Pereira C., Alsufyani N. A., Major M. P., Flores-Mir C. (2016). Accuracy and reliability of oral maxillofacial radiologists when evaluating cone-beam computed tomography imaging for adenoid hypertrophy screening: a comparison with nasopharyngoscopy. *Oral Surgery, Oral Medicine, Oral Pathology and Oral Radiology*.

[8] Abdel-Aziz M., El-Fouly M., Elmagd E. A. A., Nassar A., Abdel-Wahid A. (2019). Adenoid hypertrophy causing obstructive sleep apnea in children after pharyngeal flap surgery. *European Archives of Oto-Rhino-Laryngology*.

[9] Alhammadi M. S., Halboub E., Fayed M. S., Labib A., El-Saaidi C. (2018). Global distribution of malocclusion traits: a systematic review. *Dental press journal of orthodontics*.

[10] Ishida E., Ogawa T., Rokugo M. (2020). Management of adenoid cystic carcinoma of the head and neck: a single-institute study with over 25-year follow-up. *Head & Face Medicine*.

RETRACTED

[11] Dimberg L., Arnrup K., Bondemark L. (2015). The impact of malocclusion on the quality of life among children and adolescents: a systematic review of quantitative studies. *The European Journal of Orthodontics*.

[12] Bykova V. P. (2021). Expression of terminal deoxynucleotidyl transferase in the pharyngeal and palatine tonsils in local infectious and inflammatory diseases of the upper respiratory tract and pharynx in childhood. *Arkhiv Patologii*.

[13] Bandyopadhyay A., Slaven J. E. (2021). Health outcomes associated with improvement in mouth breathing in children with OSA. *Sleep and Breathing*.

[14] Reddy C. L., Patterson R. H., Wasserman I., Meara J. G., Afshar S. (2020). Oral and maxillofacial surgery. *Oral and Maxillofacial Surgery Clinics of North America*.

[15] Mi X., Cao Z., Wang M., Zhao H. (2021). The relationship between adenoid and tonsil hypertrophy and asthma in children and analysis of changes in asthma after adenotonsillectomy. *Lin Chung Er Bi Yan Hou Tou Jing Wai Ke Za Zhi*.

[16] Koca C. F., Erdem T., Bayındır T. (2016). The effect of adenoid hypertrophy on maxillofacial development: an objective photographic analysis. *Journal of Otolaryngology - Head & Neck Surgery*.

[17] Arsenina O. I., Piksaikina K. G., Popova A. V., Popova N. V., Perfiliev S. A., Сhistykova V. R. (2015). The effect of orthodontic treatment on the change of oropharynx features in patients with dentoalveolar anomalies and nasopharyngeal tonsil hypertrophy. *Stomatologiya (Moscow)*.

[18] Choi J. H., Kang J. H., Koh S. B., Kim N. H., Kho H. S. (2020). Development of an oral and maxillofacial frailty index: a preliminary study. *Journal of Oral Rehabilitation*.

[19] Chang A., Zhao H. (2021). Representation of specific diagnosis for low back pain using the 11th revision of international classification of diseases and related health problems: perspectives of conventional medicine and traditional medicine. *World Journal of Traditional Chinese Medicine*.

[20] Li Q., Liu R., Zhu L.-L. (2021). Quantitative evaluation of the compatibility effects of aidi injection on the treatment of hepatocellular carcinoma using targeted metabolomics: a new strategy on the mechanism study of an anticancer compound in traditional Chinese medicine. *World Journal of Traditional Chinese Medicine*.

[21] Lin S.-W., Jheng C.-H., Wang C.-L., Hsu C.-W., Lu M.-C., Koo M. (2021). Risk of dental malocclusion in children with upper respiratory tract disorders: a case-control study of a nationwide, population-based health claim database. *International Journal of Pediatric Otorhinolaryngology*.

[22] Xiang J., Liu F., Wang B., Chen L., Liu W., Tan S. (2021). A literature review on maillard reaction based on milk proteins and carbohydrates in food and pharmaceutical products: advantages, disadvantages, and avoidance strategies. *Foods*.

RETRACTED

[23] Poddębniak J., Zielnik-Jurkiewicz B. (2019). Impact of adenoid hypertrophy on the open bite in children. *Otolaryngologia Polska*.

[24] Osiatuma V. I., Otuyemi O. D., Kolawole K. A., Amusa Y. B., Ogunbanjo B. O. (2017). Dental arch dimensions of Nigerian children with hypertrophied adenoids. *Turkish Journal of Orthodontics*.

[25] Festa P., Mansi N., Varricchio A. M. (2021). Association between upper airway obstruction and malocclusion in mouth-breathing children. *Acta Otorhinolaryngologica Italica*.

